RETRACTED

# Potent Anti-Proliferative, Pro-Apoptotic Activity of the Maytenus Royleanus Extract against Prostate Cancer Cells: Evidence in *In-Vitro* and *In-Vivo* Models

**DOI:** 10.1371/journal.pone.0119859

**Published:** 2015-03-23

**Authors:** Maria Shabbir, Deeba N. Syed, Rahul K. Lall, Muhammad Rashid Khan, Hasan Mukhtar

**Affiliations:** 1 Department of Dermatology, University of Wisconsin, Madison, Wisconsin, United States of America; 2 Department of Food Science, University of Wisconsin, Madison, Wisconsin, United States of America; 3 Department of Biochemistry, Quaid-i-Azam University, Islamabad, Pakistan; National Cheng Kung University, TAIWAN

## Abstract

Prostate cancer is a leading of cause of cancer related death in men. Despite intensive investment in improving early diagnosis, it often escapes timely detection. Mortality remains high in advanced stage prostate cancer where palliative care remains the only option. Effective strategies are therefore needed to prevent the occurrence and progression of the disease. Plant-derived compounds have been an important source of several clinically useful anti-cancer agents and offer an attractive approach against prostate cancer. We previously showed that the methanol extract of Maytenus royleanus (MEM) leaves and its fractions possess significant antioxidant activity with therapeutic potential against free-radical associated damages. The present study evaluated the anti-proliferative activity of MEM in the prostate cancer model system. Analysis of MEM and its various fractions revealed the presence of triterpenoids, flavonoids and tannins, conjugated to one or more polar groups and carbohydrate moieties. Further studies against known standards established the existence of caffeic acid and quercetin 3-rhamnoside in varying concentration in different MEM fractions. Time course analysis of MEM treated prostate cancer cells indicated significant decrease in cell viability, assessed by MTT and clonogenic survival assays. This was accompanied by G2 phase arrest of cell cycle, downregulation of cyclin/cdk network and increase in cdk inhibitors. MEM treated cells exhibited cleavage of Caspase-3 and PARP, and modulation of apoptotic proteins, establishing apoptosis as the primary mechanism of cell death. Notably MEM suppressed AR/PSA signaling both in prostate cancer cell cultures and in the in vivo model. Intraperitoneal injection of MEM (1.25 and 2.5mg/ animal) to athymic nude mice implanted with androgen sensitive CWR22Rν1 cells showed significant inhibition in tumor growth and decreased serum PSA levels reciprocating in vitro findings. Taken together, our data suggest that MEM may be explored further for its potential therapeutic effects against prostate cancer progression in humans.

RETRACTED

## Introduction

In spite of progress in diagnosis and treatment, prostate cancer remains one of the most common health concerns affecting men during their lifetime. Indeed prostate cancer is the second leading cause of death among men in the United States and many Western countries [1]. Recent data project that prostate, lung, and colon cancer will account for about half of all newly diagnosed cancers in men in 2014, with prostate cancer alone accounting for about 1 in 4 cases [2].

The androgen receptor (AR) which belongs to the nuclear receptor super family plays a vital role in the development, function and homeostasis of the prostate [3]. Presence of a ligand, such as dihydrotestosterone (DHT) induces phosphorylation and conformational change in AR, resulting in its nuclear translocation, where it binds to androgen response elements on target genes and regulates transcription. Over-expression of AR and upregulation of its transcriptional activity are often observed in advanced prostate cancer [4, 5]. Androgen deprivation therapy remains the standard care for the treatment of advanced disease. Despite an initial favorable response, almost all patients invariably progress to a more aggressive, castrate-resistant phenotype. Studies on patient specimens show that the AR is expressed in nearly all cancers of the prostate, both before and after androgen ablation therapy [6]. In fact, prostate-specific antigen (PSA), which is encoded by an androgen-responsive gene, has been detected in the majority of hormone-refractory cancers, indicating that the AR signaling pathway is still functional in these cancers [7].

Screening for PSA, in combination with digital rectal examination, and needle biopsy, have improved patients’ survival by facilitating detection of early and localized disease. However, cure for the advanced and metastatic disease is still elusive [8]. Current medical treatment approaches include surgery, radiation therapy and chemotherapy, either as monotherapy or in multimodal approach [8]. The role of diet in human cancer has gained considerable attention in the last few decades and has resulted in a paradigm shift in our understanding of cancer prevention and treatment. There is emerging evidence that diet, physical activity and body weight often termed energy balance factors are important factors in modifying cancer progression, and may be linked to increased risk of cancer recurrence [9]. At present, studies are being conducted to increase our understanding of the relationship between diet and prostate cancer. Optimal nutrition can reduce the incidence of prostate cancer and may help reduce the risk of its progression. Including colorful, plant-based foods and maintaining a healthy weight have been suggested as important nutrition strategies for prostate cancer survivors [10]. A recent study showed that low prostate concentration of lycopene is linked to development of prostate cancer in patients with high-grade prostatic intraepithelial neoplasia [11]. Adherence to the Mediterranean diet comprising of abundant fruits, vegetables, legumes, nuts, unrefined cereals, olive oil and moderate quantities of fish was associated with low overall mortality after diagnosis of non-metastatic prostate cancer [12].

RETRACTED

Maytenus royleanus belongs to the family Celastraceae, a large family that comprises of approximately 100 genera and 1300 species, widely distributed in the world. Several species of Maytenus have been used in traditional medicine, for the treatment of gastrointestinal disorders, fever, arthritis etc. [13, 14]. The biological activities of Maytenus species are attributed to the presence of different classes of secondary metabolites such as phenolic glucosides, flavonoids and triterpenes [15]. In our previous studies, we showed that the methanol extract of Maytenus royleanus (MEM) leaves and its derived fractions possessed significant antioxidant activity with therapeutic potential against free-radical associated damages [15]. Here, we studied the effect of MEM on prostate cancer cell proliferation and demonstrate that MEM inhibits the growth and viability of both androgen sensitive and androgen independent prostate cancer cells and exerts potent inhibitory effect on AR/PSA signaling both in in vitro cell cultures and in vivo tumor xenografts.

## Materials and Methods

### Materials

Antibodies against cdk2, cdk4, cdk6, cyclin B1, cyclin D1, cyclin D2, cyclin E, p27, p21, PSA, Poly (ADP-ribose) polymerase (PARP), Bcl-2, Bax, Bak, Bcl-XL and AR were obtained from Cell Signaling Technology (Beverly, MA). Anti-mouse and anti-rabbit secondary antibody horseradish per-oxidase conjugate was obtained from Amersham Pharmacia Life Sciences. The Bio-Rad DC Protein Assay Kit was purchased from Bio-Rad, CA. Novex precast Tris-Glycine gels were obtained from Invitrogen. The annexin-V-FLUOS Staining Kit was purchased from Roche.

### Preparation of Plant extract

Dried leaves of MEM were first powdered followed by two extractions with 95% methanol. Filtered MEM was spray dried and suspended in 50ml distilled water and fractions were prepared in 200 ml of solvents with increasing polarity i.e., n-hexane, ethylacetate and n-butanol. Each layer was separated with vigorous shaking and the soluble leftover was used as residual aqueous fraction.

RETRACTED

### Phytochemical screening

#### [A] Liquid chromatography mass spectrometric analysis

MEM was analyzed by LC-MS to generate a fingerprint of phytochemicals present in the plant. Dried sample of MEM and its various fractions were dissolved in 15mg/ml of methanol. Undissolved particles were removed and 10μl of the sample was subjected to HILIC chromatography in negative ionization and reverse phase (RP) both in positive and negative ionization modes to target flavonoids and phenolic acids. For HILIC separation, samples were chromatographically resolved with Phenomenex Luna HILIC, 3μm, 2x150mm column on Agilent 1200 HPLC (Agilent, CA) with an auto-sampler held at 5°C, using linear gradient of 10mM ammonium formate (pH = 4.5) in water and 1mM ammonium formate (pH = 4.5) in 99% acetonitrile over 45 minutes. For positive RP separation, samples were chromatographically resolved with Agilent ZORBAX 300SB-C18, 1.8μm, 2.1x50mm column on an Agilent 1200 HPLC (Agilent, Palo Alto, CA) with an auto-sampler held at 5°C, using linear gradient of 0.1%Formic acid in water and 0.1% formic acid in acetonitrile over 60 min. For negative RP separation, similar instrument setup for positive mode was used as above while changing the mobile phase to a linear gradient of 10mM ammonium formate (pH 6.5) in water and 1mM ammonium formate (pH 6.5) in 99% acetonitrile over 45 minutes. The flow rate for both the separation modes was 250μl/min.

#### [B] High performance liquid chromatography (HPLC) of plant extract

250 mg of plant powder was extracted with 10 ml of 25% HCl and 25 ml of chloroform. The extract was filtered and diluted to 100ml. 10μl of filtered samples were injected into the Agilent 1200 HPLC system. Separation was carried out through a C18 column equipped with a UV-VIS Spectra-Focus detector, injector and auto sampler). Trifluoroacetic acid and acetonitrile were used as mobile phases with flow rate of 1ml/min. Caffeic acid and quercetin 3-rhamnoside were used as internal standards for comparative detection within the MEM fractions. The calibration curves were generated for both standard compounds in the range of sample quantity (0.02–0.5 μg). All runs were done in triplicate.

### Treatment of cells

C_4-2_ and CWR22Rν1 human prostrate carcinoma cells were purchased from ATCC (American type culture collection). Both cell lines were grown in RPMI 1640 (Life Technologies, NY) supplemented with 10% FBS and 1% penicillin/streptomycin, with 5% CO_2_, at 37°C. MEM dissolved in DMSO was used for the treatment of cells. Cells at a confluency of ~70% were treated with MEM at 10–100μg/ml for 24h in complete cell medium where the final concentration of DMSO used for each treatment was less than 0.1% (v/v).

RETRACTED

### Cell viability assay

3-(4,5-dimethylthiazol-2-yl)-2,5-diphenyl tetrazoliumbromide (MTT) assay was employed to study the effect of MEM on the viability of C_4-2,_ PC3, DU145 and CWR22Rν1cell lines. The cells were plated (1×10^4^ cells per well) in 1ml of complete culture medium containing 10–200μg/ml concentrations of MEM in 24-well microtiter plates. After incubation in a humidified incubator for 24h at 37°C, 200μl of MTT (5mg/ml:1XPBS) was added to each well and incubated for two hours, after which 200μl of DMSO was added. The plates were then centrifuged (1800×g for 5min at 4°C). The absorbance at 540nm was recorded on a microplate reader. The effect of MEM on growth inhibition was calculated as % cell viability where DMSO-treated cells were taken as 100% control.

### Clonogenic assay

The effect of treatment on clonogenic survival of prostate cancer cells was determined using colony formation assay. Both CWR22Rν1 and C_4-2_ cells were treated with increasing concentrations (20, 40 & 60μg/ml) of MEM in RPMI-1640 complete medium. Following treatment, the cells were re-plated in triplicate on a 6-well tissue culture plate with 5000 cells/well and cultured in 5% CO2 at 37°C for 8 days with growth media being replaced with/without MEM every 2 days. The cells were then stained with 0.5% crystal violet (in methanol: H_2_O; 1:1) and pictures were taken using a digital camera. The pictures were enhanced using Adobe Photoshop for brightness, contrast, and sharpened for uniformity of appearance.

### Cell cycle analysis/apoptosis by flow cytometry

CWR22Rν1 and C_4-2_ cells treated with MEM (20–60μM:24h) in complete medium were trypsinized and fixed in 1% Paraformaldehyde:1XPBS for an hour and washed twice with cold PBS and centrifuged. The pellet was suspended in chilled 70% ethanol and stored overnight. Next, the cells were centrifuged for 5min at 1000 rpm, and the pellet obtained was washed twice with cold PBS to remove ethanol. The cells were labeled with FITC and propidium iodide using the Apo-Direct Kit (BD Pharmagen, CA) as per manufacturer’s protocol. Analysis was performed with a FACScan (Becton Dickinson, NJ). About 10,000 cells per sample were collected and the DNA histograms were analyzed with ModFitLT software (Verily Software House, ME).

### Protein extraction and Western blot analysis

After treatment with MEM ice-cold lysis buffer was added to the cells (50nmol/liter Tris-HCl,150mmol/liter NaCl, 1 mmol/liter EGTA, 1 mmol/liter EDTA, 20 mmol/liter NaF,100 mmol/liter Na3VO4, 0.5% Nonidet P-40, 1% Triton X-100, 1 mmol/liter PMSF, pH 7.4) with protease inhibitors (Calbiochem, Germany) incubated over ice for 20min. For western blotting 8–12% poly acrylamide gels were used to resolve 40μg of protein, transferred on to a nitrocellulose membrane, probed with appropriate monoclonal primary antibodies, and detected by chemiluminescence autoradiography after incubation with specific secondary antibodies.

RETRACTED

### Gene expression analysis

Total RNA was isolated from cells using a commercial RNeasy kit (Qiagen, CA) RNA concentration was measured spectrophotometrically at 260nm and cDNA was made, following the manufacturer protocol. The reaction mixture was prepared containing 10μL FastStart Universal SYBR green Master (Roche, Germany), 6μM reverse primers, and 10μg cDNA, with RNAase free water added to a total volume of 20μL. The amplification and real time analysis was done for 40 cycles with following factors; 95°C (10min) in order to activate of Fast Start Taq DNA polymerase; 60°C (1min) for amplification and real time analysis. The gene expression levels were determined using 2^-ΔΔCT^. Primer sequence used were; AR Sense 5’-CTGGACACGACAACAACCAG-3’; AR Antisense 5’- CAGATCAGGGGCGAAGTAGA-3’; GAPDH Sense 5’-AAGGTCGGAGTCAACGGATTTGGT-3; GAPDH Antisense 5’-ACAAAGTGGTCGTTGAGGGCAATG-3’.

### Imunofluorescence microscopy

C_4-2_ and CWR22Rν1 cells were seeded on a two-chamber tissue culture glass slides and treated with 40μg/ml of MEM at 70% confluence for 24h. After washing with PBS cells were fixed with 2% paraformaldehyde followed by permeabilization with methanol and blocking with 2% serum. Incubation with primary antibodies overnight was followed by incubation with appropriate fluorophore tagged secondary antibodies. Antifade DAPI (Invitrogen, NY) was used as mounting and counterstaining medium. For analysis, Bio-Rad Radiance 2100 MP Rainbow system for biological imaging was used. To detect apoptotic and necrotic cells the Annexin-V-Fluos Staining Kit (Roche, Switzerland) was used according to the manufacturer’s protocol. Zeiss LSM 410 confocal microscopy was used to measured fluorescence. The cells stained with Annexin-V and unstained cells in a selected field were counted to ascertain the extent of apoptosis and necrosis.

### PSA ELISA

For quantitative determination of PSA levels in the C_4-2_ and CWR22Rν1 cells human PSA ELISA kit (Anogen, Ontario, Canada) was used according to the manufacturer’s protocol.

### Ethical Statement for animal studies

Athymic nude mice studies were conducted according to the Institutional guidelines for the care and use of animals and were approved by Animal Care and Use Committee, School of Medicine and Public Health, University of Wisconsin-Madison.

### In vivo tumor xenograft model

Athymic (nu/nu) male nude mice obtained from NxGen Biosciences (San Diego, CA) were housed under pathogen-free conditions (12h light/12h dark schedule) and fed with an autoclaved diet adlibitum. We selected CWR22Rν1 cells for determining the in vivo effects of MEM as these cells form rapid and reproducible tumors in nude mice. The implantation of CWR22Rν1 cells is also responsible for secretion of significant amounts of PSA in the blood stream of the host. Tumor xenografts in mice were established by subcutaneous injection of CWR22Rν1 cells (1×10^6^) mixed with Matrigel (Collaborative Biomedical Products, MA) in a ratio of 1:1. Eighteen animals were randomly selected into three groups consisting of six animals each. The first group of animals serving as control group received DMSO intra-peritoneally (i.p). The animals of groups 2 and 3 received i.p. injection of MEM, 1.25mg and 2.5 mg per animal, respectively, twice weekly and throughout the study body weight, diet, and water consumption were recorded. Tumor volume was calculated by the formula 0.5238×L1×L2×H (L1 = long diameter, L2 = short diameter, and H = height of the tumor) and tumor sizes were measured twice weekly. Animals were euthanized using CO2 inhalation method following ARAC guidelines, when tumor volumes reached to ~1200mm^3^. Blood samples were collected by the mandibular bleed and serum separated from the whole blood was stored at −20°C. Serum PSA levels were assayed by the PSA ELISA kit described above. H&E stained slides of lung, kidney, liver, heart and brain were prepared to examine the possible toxic effects of MEM treatment.

RETRACTED

### Immunohistochemistry

Tumor tissues sections were stained with hematoxylin and eosin for morphological visualization. Moreover, tissues fixed in 10% formalin were subjected to immunohistochemical analysis. Briefly, after deparaffinization in sodium citrate buffer, sections were incubated overnight with antibodies against cleaved Caspase-3 and Histone 3-phosphate (H3-P) [1:75] (Cell Signaling, MA) followed by incubation with appropriate HRP-conjugated secondary antibodies, diamminobenzidine/DAB (DAKO, CA) staining and counter staining with hematoxylin. After mounting with Permount, sections were covered with cover slips and staining was analyzed by an experienced pathologist blinded to treatment groups.

### Statistical Analysis

All statistical analysis was carried out with GraphPad prism (San Diego, CA) and p values <0.05 were considered significant.

## Results

### Phytochemical analysis of MEM

MEM along with n-hexane, butanol, ethyl acetate and residual aqueous fractions were separated by LC-MS analysis. This technique was primarily used to generate a fingerprint of the phytochemical composition of the MEM. The extract seems to be a complex mixture of unknown phytochemicals as seen in the base peak chromatogram of the HILIC (-ve) chromatogram (Fig. 1). The HILIC run of MEM showed the presence of 164 compounds based on base peaks generated from molar mass and retention time of compounds (Fig. 1A; data attached as S1_Dataset). Extending the same data analysis to the other fractions in HILIC (-ve) mode, the n-butanol fraction contained 79 compounds while the ethyl acetate and n-hexane fractions showed 69 and 40 compounds respectively. C18 RP (-ve) chromatogram of residual aqueous fraction showed the presence of 84 compounds while the HILIC (-ve) showed 83 compounds. Based on the preliminary evidence obtained from the LC-MS data, outlined above (Fig. 1A), further analysis was performed to categorize the constituent compounds of MEM, using UV-diode array detectors. Caffeic acid and quercetin-3-rhamnoside were identified by comparing their UV and MS spectra to the corresponding internal standards. UV spectra of n-hexane, ethylacetate and n-butanol fractions revealed the presence of caffeic acid and quercetin-3-rhamnoside in varying concentrations indicating that MEM has a high content of flavonoids with known anti-cancer activity (Fig. 1B; S1 Fig).

RETRACTED

**Fig 1:** Phytochemical fingerprint of MEM. **a.** Table showing total number of compounds found in MEM and its various fractions with HILIC and C18 RP chromatography, based on retention time and molar mass; Total ion chromatograms of various fractions: ethyl acetate fraction (-ve HILIC); n-butanol fraction (-ve HILIC); n-hexane fraction (-ve HILIC); aqueous fraction (-ve HILIC); aqueous fraction (-ve C18 RP). **b.** UV chromatograms of ethyl acetate n-hexane and n-butanol fractions of MEM, at 280, 320 & 370 nm, with caffeic acid and quercetin 3-rhamnoside internal standards.

### MEM inhibits growth and viability of prostate cancer cells

Since both these compounds are known to possess anti-cancer activities, we asked whether the extract itself would be more effective in inhibiting the growth and viability of prostate cancer cells. To investigate the anti-proliferative potential of MEM, we performed 3-(4, 5-dimethythiazol-2-yl)-2, 5-diphenyl tetrazolium bromide (MTT) assay against androgen-sensitive (C_4-2_ and CWR22Rν1) and androgen-independent (PC3 and DU-145) prostate cancer cells. We observed that MEM treatment (10–180μg/ml for 24h and 48h) to prostate cancer cells caused inhibition of cell growth in a dose-dependent manner. Time course analysis revealed that there existed only a modest difference between the decrease in cell viability of cells at 24h and 48h, suggesting that prostate cancer cells respond to MEM treatment within 24h. As shown in (Fig. 2A), the IC_50_ values of MEM-treated CWR22Rν1 were 47.4 &42 μg/ml; for C_4-2_, 52.8& 44.4 μg/ml; for PC3, 61.8 & 36 μg/ml; and for DU145, 90.6 & 88.2 μg/ml for 24 and 48h respectively. The data suggested that androgen-sensitive C_4-2_ and CWR22Rν1 cells showed slightly better sensitivity to MEM treatment than DU145 and PC3cells (Fig. 2A). Clonogenic assay further validated these findings where CWR22Rν1 and C_4-2_ cells treated for seven days with MEM at 20, 40 & 60 μg/ml showed a significant dose-dependent inhibition of colony formation relative to untreated controls (Fig. 2B). The different fractions of MEM separated on the basis of polarity in different solvents like n-hexane, ethylacetate, n-butanol and water were also investigated for their growth inhibitory effect on CWR22Rν1 cells. The n-hexane and aqueous fractions proved to be more potent in inhibiting proliferation of CWR22Rν1 cells (20 & 36μg/ml) as compared to the butanol and ethylacetate fractions (39.6 & 66.8μg/ml) (Fig. 2C).

RETRACTED

**Fig 2:** MEM inhibits growth and viability of prostate cancer cells. a. Prostate cancer cells were treated with MEM for 24/48h, and cell viability was determined by MTT assay. Table shows the IC_50_ of *CWR*22Rν1, C_4-2_, PC-3 and DU145 at 24 and 48h. Mean ± SD of experiments performed in triplicate is shown. **b.** Dose-dependent effect of MEM on clonogenecity of *CWR*22Rν1 and C_4-2_ cells as detected by colony formation assay. Details are described in material methods. **c.** Effect of various fractions (n-hexane, ethyl acetate, n-butanol and aqueous) on viability of *CWR*22R ν1 cells, determined by MTT assay. *p<0.05 and **p<0.01 was considered statistically significant.

### MEM induces G2 phase arrest of prostate cancer cells

To assess the cell cycle profile of MEM-treated prostate cancer cells we performed flow cytometric analysis and observed the effect of MEM on cell cycle distribution. A significant dose-dependent increase in cell population in the G2 phase of the cell cycle was observed as a result of MEM treatment in CWR22Rν1 and C_4-2_ cells. The G2 phase cell cycle distribution for C_4-2_ was 25.7%, 44.61%, 59.52% and for CWR22Rν1was 38.6%, 47.72%, and 57.72% at 20, 40 and 60μM concentrations of MEM respectively (Fig. 3A; S2 Fig). The increase in G2 phase cell population was accompanied by a simultaneous decrease in the G0/G1 and S phase cell population. We next examined the effect of MEM on cell cycle regulatory molecules operative in the G2 phase of the cell cycle. Immunoblot analysis showed that MEM treatment to C_4-2_ and CWR22Rν1 resulted in decreased protein expressions of cdks 2, 4 & 6 and cyclins B1, D1, D2 & E compared to the untreated controls (Fig. 3A and 3B; S3 Fig). This was associated with noticeable induction of p21 and p27 in MEM treated cells (Fig. 3D; S3 Fig).

RETRACTED

**Fig 3:** MEM induces G2 phase arrest of prostate cancer cells. a. *CWR*22Rν1 and C_4-2_ cells treated with MEM for 24h were stained with propidium iodide and analyzed by flow cytometry. Percentage of cell population in G2-phase of the cell cycle is shown in the box of each histogram. Mean ± SD of experiments performed in triplicate is shown. **b-d.** Effect of MEM treatment on cell cycle regulatory proteins: Whole cell lysates of *CWR*22Rν1 and C_4-2_ cells with/without MEM (20–60 μg/ml: 24h) were subjected to SDS-polyacrylamide gel electrophoresis. Equal loading was confirmed by reprobing with GAPDH. The immunoblots shown are representative of three independent experiments with similar results.

### MEM induces apoptosis through activation of intrinsic and extrinsic pathway

To examine whether the observed decrease in cell viability is linked to induction of apoptosis we performed Annexin staining of MEM treated prostate cancer cells. We used Annexin V tagged to FITC, which has a strong and specific affinity for phosphatidylserine, to monitor its translocation to the plasma membrane. MEM treated cells showed a significant increase in green fluorescence in contrast to untreated controls indicating that treatment with MEM induced apoptosis in prostate cancer cells (S4 Fig). Flow cytometric analysis was then performed to quantify the number of cells undergoing apoptosis as a result of MEM treatment. A significant dose-dependent increase in the population of apoptotic cells was observed in both cell lines, a result of MEM treatment (Fig. 4A; S4 Fig). Immunoblot analysis was employed next to study the expression of proteins involved in cellular apoptosis. Caspase-3, a member of the Caspase family of aspartate-specific cysteine proteases plays a central role in the execution of the apoptotic program. PARP-1 is one of several known cellular substrates of Caspases and cleavage of PARP-1 by Caspases is considered to be a hallmark of apoptosis [16]. MEM treated cells showed increased expression of activated Caspase-3; associated with PARP cleavage (Fig. 4B; S5 Fig) further validating that apoptosis is the primary mechanism of MEM-induced cell death. To investigate whether MEM induced apoptosis is mediated through activation of intrinsic or extrinsic pathways we next studied the expression of Caspases -8 and -9 in MEM treated cells. We found an induction of cleaved Caspase-8 in cells treated with 20, 40 and 60 μg/ml of MEM (Fig. 4C; S5 Fig). Concomitant decrease in the pro-form of Caspase-9 and Bid in CWR22Rν1 and C_4-2_ cells, post MEM treatment suggested activation of both extrinsic and intrinsic pathways of apoptosis. We assessed the effect of the extract on the Bcl-2 family of proteins, involved in apoptosis. MEM treated cells showed an increase in the expression of pro-apoptotic Bax and Bak and a decrease in the expression of anti-apoptotic Bcl-2 and Bcl-X_L_ proteins (Fig. 4D; S5 Fig).

RETRACTED

**Fig 4:** MEM induces apoptosis through activation of intrinsic and extrinsic pathway. a. *CWR*22Rν1 and C_4-2_ cells treated with MEM (20–60 μg/ml: 24h) were labeled with FITC and analyzed by flow cytometry. Percentage of apoptotic cells with the corresponding dose of MEM is shown in each histogram. Mean ± SD of experiments performed in triplicate is shown. **b-d.** Whole cell lysates of *CWR*22Rν1 and C_4-2_ cells with/without MEM (20–60 μg/ml: 24h) treatment were subjected to SDS-polyacrylamide gel electrophoresis. Effect of MEM treatment on proteins involved in apoptosis pathways. Equal loading was confirmed by reprobing with GAPDH. The immunoblots shown are representative of three independent experiments with similar results.

### MEM decreases AR and PSA expression in prostate cancer cells

Androgens play an important role in development and progression of prostate cancer and PSA, a well-known androgen-responsive gene is currently the most accepted marker for assessment of prostate cancer progression in humans [17]. The effect of MEM treatment on AR and PSA expression was examined in CWR22Rν1and C_4-2_ cell lines employing immunoblotting and RT-PCR. A significant decrease in AR protein expression was observed with MEM treatment (Fig. 5A and 5B; S6 Fig). Immunofluorescence staining of CWR22Rν1 & C_4-2_ cells showed decrease nuclear localization of AR in MEM treated cells as compared to control (Fig. 5B).The CWR22Rν1 and C_4-2_ prostate cancer cells exhibit high protein levels of intracellular PSA, as evidenced by a 34-kDa PSA band (Fig. 5A). The dose dependent effect of MEM on CWR22Rν1 and C_4-2_ cells resulted in a significant decrease in PSA protein levels at 20, 40 and 60 μg/ml concentrations (Fig. 5A; S6 Fig). The decrease in protein expression was accompanied by reduced transcript levels of AR in MEM treated cells (Fig. 5C; S6 Fig). We further determined the secreted PSA levels in CWR22Rν1 and C_4-2_ cell lines, employing the quantitative sandwich ELISA technique. A significant reduction in PSA levels was noted in both cell lines with MEM (40 μg/ml) treatment (Fig. 5D).

**Fig 5:** MEM decreases AR and PSA expression in prostate cancer cells. a. Whole cell lysates of *CWR*22Rν1 and C_4-2_ cells with/without MEM (20–60 μg/ml: 24h) were subjected to SDS-polyacrylamide gel electrophoresis. Equal loading was confirmed by reprobing with GAPDH. The immunoblots shown are representative of three independent experiments with similar results. **b.** Immunofluorescence microscopy with Alexa fluor staining of AR (green fluorescence) in *CWR*22Rν1 and C_4-2_ cells, counter stained with DAPI (blue fluorescence). **c.** qPCR analysis of MEM treated *CWR*22Rν1 and C_4-2_ cells for changes in AR mRNA levels. The data expressed as fold change represent the mean±standard errors experiments performed in triplicates where *p < 0.05, **p < 0.01 was considered significant vs control. **d.** Effect of MEM on secreted levels of PSA in *CWR*22Rν1 and C_4-2_ cells treated with MEM (40 μg/ml: 24h). PSA levels were determined by ELISA, as described in Materials and Methods; the figures represent the data of three experiments, each conducted in duplicate, where ^*p<0.05 MEM treated vs DMSO treated control cells was considered significant. **e.** Effect of MEM on DHT stimulated protein expression of AR and PSA: Whole cell lysates of *CWR*22Rν1 and C_4-2_ cells treated with MEM (40 μg/ml: 24h) were subjected to SDS-polyacrylamide gel electrophoresis. Equal loading was confirmed by reprobing with GAPDH. The immunoblots shown are representative of three independent experiments with similar results.

RETRACTED

Since DHT is known to stabilize AR protein in target cells, we next examined whether MEM by antagonizing the effect of DHT could destabilize AR protein in CWR22Rν1 and C_4-2_ cells. Both cell lines were grown in (hormone free) charcoal stripped serum containing media with 5nmol/L of DHT. Low AR protein expression was observed in untreated cells as compared to cells treated with DHT which exhibited increased AR levels. Co-treatment with DHT and MEM (40 μg/ml) for 24 hours resulted in decreased expression of AR and PSA proteins signifying that MEM functionally antagonizes DHT mediated AR stabilization (Fig. 5E; S6 Fig). Hence, the effects of MEM on AR/PSA signaling correlate with growth inhibition and cell cycle arrest of prostate cancer cells.

### MEM inhibits growth of CWR22Rν1xenografts in athymic nude mice

Given the significant inhibitory effect of MEM on AR signaling in the in vitro cell culture system, we next evaluated its efficacy *in an in vivo* model. CWR22Rν1 tumor xenografts were implanted subcutaneously in the athymic nude mice and the effect of MEM was evaluated employing two doses (1.25mg and 2.5mg/ animal). MEM was administered i.p. to these animals twice a week starting a week after tumor implantation. Appearance of small solid tumors was observed at day 8 of cell inoculation in DMSO treated nude mice. This period was prolonged to 15–18 days in MEM treated animals. Significant decrease in tumor growth was observed in MEM treated group, as compared to the treated controls (Fig. 6A). Thus, in animals of control group the average tumor volume of 800 mm^3^ was reached in ~ 36±3 days after tumor cell inoculation. At the same time point, the average tumor volumes of the 2.5mg and 1.25mg MEM treated groups were 56 and 74mm^3^ respectively (Fig. 6A). Tumor sections of treated and control groups were evaluated using H&E staining and immunohistochemistry (Fig. 6B). To assess in vivo inhibition of AR signaling to diminished tumor growth, upon MEM administration, we analyzed the expression of AR, apoptosis (Caspase-3) and proliferative (H3-P) markers, in the tumor sections. Intense nuclear staining of AR was significantly absent in MEM treated samples. Immunoblot analysis of tumor tissue lysates demonstrated significant downregulation of AR and PSA protein expression in MEM treated animals. The serum PSA levels were similarly decreased in MEM treated animals (Fig. 6C; S7 Fig). Immunostaining for H3-P showed remarkably low immune-reactivity in MEM treated animals compared to the controls. In contrast, tumor sections from MEM-treated groups showed an increase in cleaved Caspase-3 staining, further corroborated by immunoblot studies. Western blot data demonstrated reduced Ki-67 expression in MEM treated tumors, another established marker of cell proliferation (Fig. 6D; S7 Fig).

RETRACTED

**Fig 6:** MEM inhibits growth of *CWR*22Rν1xenografts in athymic nude mice. **a.** Average tumor volume of DMSO, 2.5mg & 1.25mg MEM injected mice plotted over days after *CWR*22Rν1 tumor xenografts implanted in athymic nude mice. Values represent mean±SE of six mice, where MEM (1.25mg) *^p<0.05 and MEM (2.5mg) *p<0.01 versus DMSO treated control was considered significant. **b.** Top panel: H&E staining of MEM treated xenograft tumor tissue vs control. Immunohistochemical analysis of AR in MEM treated tumor tissue vs untreated control. Bottom panel: Whole cell lysates of tumor xenografts from animals treated with/without MEM were subjected to SDS-polyacrylamide gel electrophoresis. Equal loading was confirmed by reprobing with GAPDH. The immunoblots shown are representative of three independent experiments with similar results. **c.** Serum PSA levels of MEM treated mice were analyzed by ELISA, as described in Materials and Methods. MEM (1.25mg) and MEM (2.5mg) *p<0.01 versus DMSO treated control was considered significant. **d.** Top panel: Immunohistochemical analysis of H3P & cleaved caspase 3 in MEM treated tumor tissue vs untreated control. Bottom panel: Whole cell lysates of tumor xenografts from animals treated with/without MEM were subjected to SDS-polyacrylamide gel electrophoresis. Equal loading was confirmed by reprobing with GAPDH. The immunoblots shown are representative of three independent experiments with similar results.

RETRACTED

### MEM treatment is not associated with adverse side effects

Since toxicity of the extract was a major consideration, body weights were recorded twice a week to evaluate the general health and well-being of animals during treatment. As shown in (Fig. 7A), no significant weight changes were observed in the treated versus the control groups. Moreover, the animals displayed no signs of discomfort during the treatment regimen. The histopathological evaluation of the tissues of lung, liver, brain, heart, and kidneys from both vehicle- and MEM- treated mice revealed no detectable differences in architecture (Fig. 7B and 7C). No signs of toxicity, specific to MEM treatment, were detected in the organs by the pathologist (S1_Pathologist Report). However, the liver of some animals from both treated and control groups, displayed mild inflammation suggestive of peritonitis. Collectively, the data generated from xenograft studies strongly suggested induction of robust apoptosis associated with tumor growth inhibition and suppressed AR/PSA signaling in MEM treated mice with no adverse effects associated with the treatment.

**Fig 7:** MEM treatment is not associated with adverse side effects. **a.** Mice weight was taken twice weekly and values represent mean±SD of six mice. (B&C) H&E staining was performed for toxicity studies on heart, brain, lung, kidney and liver tissues of mice treated with DMSO or MEM.

## Discussion

A variety of factors including inflammation, antioxidant deficiency, compromised immune system, nutrient deficiencies and genetic predisposition are thought to predispose to cancer [18]. There is strong scientific evidence indicating that regular consumption of fruits and vegetables is negatively associated with the risk of developing cancer [19–22]. The presence of a wide range of phytochemicals in plants and vegetables is presumably Mother Nature’s design to confer optimal health benefits to living beings including humans. Since carcinogenesis is a multistage process, it is unlikely that a single agent could serve to combat this dreaded disease. Thus the synergistic interactions between the phytonutrients present in a plant based extract may help protect against cancer. Lack of toxicity and easy acceptance are additional benefits of naturally occurring compounds [23].

In recent years, plant-based extracts have been subjected to rigorous fractionation in an effort to identify their active ingredients. However, there is reason to believe that the beneficial effects of whole foods may overshadow those from isolated nutrients. In this context, certain fractions of whole extracts enriched in phytochemicals such as polyphenols, carotenoids and anthocyanins have shown greater efficacy than their isolated ingredients. For example, the beneficial effects of pomegranate have been attributed to the presence of flavonoids, anthocyanidins, ellagic acid, ellagitannins (including punicalagins), punicic and other fatty acids which seem to be its most therapeutically effective components [24]. Studies examining the complex interplay between the phytochemicals present in pomegranate support the concept of supra-additive anticancer effect of these compounds [25–27]. The synergistic effect of its constituents appears to be superior when compared to individual constituents [24]. Similar studies using extracts from other fruits or plants have shown that the chemical synergy of the constituents is more effective in terms of anti-carcinogenic activity than individual or purified ingredients [28]. This may be a result of inhibition of multiple targets at the same time with subsequently greater likelihood for producing cancer protective effects.

RETRACTED

We have focused our attention on a plant Maytenus royleanus that has been used successfully in traditional medicine for the treatment of gastrointestinal disorders, fever, arthritis etc. In our previous published study, we reported that the methanolic extract of the plant leaves, (referred as MEM) possesses significant anti-oxidant activity as evidenced by results of various antioxidant assays employed in our study [15]. Qualitative analysis of MEM showed the presence of alkaloids, anthraquinones, cardiac glycosides, coumarins, flavonoids, saponins, phlobatannins, tannins and terpenoids [15]. MEM and its derived fractions also displayed anti-lipid peroxidation efficacy against free-radical associated damages and anti-hemolytic properties. These findings emphasized the therapeutic potential of MEM, likely attributable to the high concentration of phenolic flavonoid, tannins and terpenoids [15]. However, the flavonoid components of MEM remain undefined. In the present study, employing quantitative HPLC and MS techniques we identified caffeic acid and quercetin-3-rhamnoside as two principal flavonoids present in MEM. Both compounds possess a wide spectrum of pharmacological potential such as anti-oxidant, anti-inflammatory activities and their anti-cancer effect is currently being explored [29–31].

We therefore proceeded to examine the molecular basis of the anti-cancer activity of the phytochemical rich MEM extract against prostate cancer cells, in vitro and in vivo. Our data demonstrate that MEM treatment of human prostate cancer CWR22Rν1 and C_4-2_ cells resulted in cell growth arrest, alteration in molecules regulating cell cycle operative in the G2 phase of the cell cycle and apoptosis in a dose dependent manner (Fig. 3 and 4). A major underlying cause of cancer development is attributed to accelerated or dysregulated proliferation leading to cellular expansion and accumulation of tissue mass. In eukaryotes, transit through the cell cycle is coordinated by a family of protein kinase complexes, comprised of a catalytic subunit, the cyclin dependent kinase and its activating partner, cyclin [32, 33]. Association of cyclins B1 and D with cdks 2, 4 or 6 in a controlled cell growth environment causes phosphorylation of RB and its release from E2F which results in progression of the cell cycle and cellular growth [32, 34, 35]. Our results showed decreased expression of cyclins B, D and E and cdks 2, 4 and 6 accompanied with an increase in expression of cdk inhibitors WAF1/p21 and KIP1/p27 in MEM treated cells. Moreover, MEM treated prostate cancer cells displayed arrest in the G2 phase of the cell cycle (Fig. 3). These are important findings because cell cycle regulation is an important target for prevention against prostate cancer.

RETRACTED

Dysregulated cell cycle, with subsequent impact on elements of proliferative control such as cell cycle checkpoints and the response to DNA damage is only part of the problem in cancer treatment [36]. Recent investigations in the field of tumor biology have broadened our understanding to encompass aberrant cellular survival, and failure to induce apoptosis or cell death, as a major contributor to the transformed state. For that reason, many current chemotherapeutic strategies are designed to trigger tumor-selective cell death with limited detrimental effect to normal cell function [37]. MEM treatment was shown to activate the extrinsic and the intrinsic apoptotic pathways with subsequent cleavage and inactivation of PARP (Fig. 4B and 4C). Bcl-2, an apoptosis suppressor, and an upstream effector in the apoptotic pathway, is highly expressed in a majority of human tumors. Bcl-2 forms a heterodimer complex with Bax, neutralizing the pro-apoptotic effects of the latter [34]. Our data suggest that MEM mediated increase in the expression Bax and down regulation of Bcl-2 may be a possible route through which MEM induces apoptosis in prostate cancer cells (Fig. 4D). In addition, MEM was able to target Bcl-xl and Bak indicating its pleiotropic effect on the apoptotic signaling pathway (Fig. 4D).

The AR signaling remains a fundamental component in the development of normal prostate tissue and also in the progression of prostate cancer [38]. Recent work has shown that castration resistant prostate cancers continue to depend on AR signaling which is reactivated despite low serum androgen levels [39]. In addition, currently available AR targeted therapy, including GnRH agonists and anti-androgens, cannot completely shut down AR signaling [40]. Based on the current knowledge of the biologic drivers of prostate cancer progression, it is reasonable to assume that androgen deprivation in prostate cancer at an early stage when it is most sensitive to androgen stimulus may produce better and more durable disease responses, resulting in prolonged survival and delayed progression to the resistant stage. This suggests that finding new methods to impede AR signaling might considerably improve the benefits of therapeutic strategies used for the cure of the disease [41–43]. MEM treated CWR22Rv1 and C_4-2_ cells showed decreased AR expression both at protein and mRNA levels, associated with inhibition of AR-specific PSA (Fig. 5). Furthermore, in our studies, DHT exposed cells co-treated with MEM displayed a marked inhibition in AR and PSA protein expression presumably due to AR mediated decrease in AR stability and down regulation in AR gene transcription. We verified our in vitro findings in an in vivo model where athymic nude mice were injected with androgen responsive CWR22Rν1 cells that secrete PSA in the blood stream of the host. Similar to our in vitro data, i.p. injection of MEM considerably slowed tumor growth in athymic mice (Fig. 6A), inhibited AR expression and resulted in a significant decrease in the serum PSA levels (Fig. 6B and 6C). No significant change in the tissue architecture, decrease in body weights and other associated adverse effects in mice treated with MEM (Fig. 7) further supported the notion that the extract may be a potential addition in the arsenal of naturally derived agents, currently being explored for the prevention and treatment of prostate cancer. Taken together, the present study could have a useful implication and translational significance to prostate cancer patients as it shows that MEM can inhibit tumor progression, which could increase the survival and quality lifespan of the patients suffering with prostate cancer.

RETRACTED

## Supporting Information

S1 Fig Effect of Caffeic acid and Quercetin on growth and viability of prostate cancer cells. *CWR*22Rν1 cells were treated with Caffeic acid, Quercetin 3-rhamnoside and Caffeic acid + Quercetin 3-rhamnoside for 24h, and cell viability was determined by 3-(4,5-dimethylthiazol-2-yl)2,5diphenyltetrazoliumbromide assay. Data shown are mean ±SD of three separate experiments, where *p<0.05, **p<0.01, ***p<0.001 vs. control were considered statistically significant.
(TIF)

S2 Fig *CWR*22Rν1 and C_4-2_ cells treated with MEM (0–60 μg/ml: 24h) were stained with propidium iodide and analyzed by flow cytometry. Percentage of cell population in various phases of the cell cycle is tabulated. Mean ± SD of experiments performed in triplicate is shown.
(TIF)

S3 Fig Whole cell lysates of *CWR*22Rν1 and C_4-2_ cells with/without MEM (20–60 μg/ml: 24h) treatment were subjected to SDS-polyacrylamide gel electrophoresis to evaluate the effect on cell cycle regulatory proteins. Equal loading was confirmed by reprobing with GAPDH. Densitometric analysis of immunoblots from three independent experiments was performed using Image J after normalizing to GAPDH; values plotted for each protein are shown in respective histograms. +*p<0.05 vs. control was considered statistically significant.
(TIF)

S4 Fig Effect of MEM treatment on cell growth and apoptosis. a. Fluorescence microscopy was performed to evaluate apoptosis in MEM (40 μg/ml: 24h) treated *CWR*22Rν1 cells. Apoptotic cells were stained green with Annexin-V while necrotic cells stained red with propidium iodide. Details are described in materials and methods. b. After 24h treatment with MEM (0–60 μg/ml: 24h) *CWR*22Rν1 and C_4-2_ cells were incubated with FITC and analyzed by flow cytometry. Percentage of apoptotic cells is tabulated.
(TIF)

S5 Fig Whole cell lysates of *CWR*22Rν1 and C_4-2_ cells with/without MEM (20–60 μg/ml: 24h) treatment were subjected to SDS-polyacrylamide gel electrophoresis to evaluate the effect on apoptosis markers. Equal loading was confirmed by reprobing with GAPDH. Densitometric analysis of immunoblots from three independent experiments was performed using Image J after normalizing to GAPDH; values plotted for each protein are shown in respective histograms. +*p<0.05 vs. control was considered statistically significant.
(TIF)

S6 Fig Effect of MEM treatment on AR and PSA. a. Whole cell lysates of *CWR*22Rν1 and C_4-2_ cells with/without MEM (20–60 μg/ml: 24h) were subjected to SDS-polyacrylamide gel electrophoresis, and effect of treatment was evaluated on AR and PSA protein levels. Equal loading was confirmed by reprobing with GAPDH. Densitometric analysis of immunoblots from three independent experiments was performed using Image J after normalizing to GAPDH; values plotted for each protein are shown in respective histograms. +*p<0.05 vs. control was considered statistically significant. b. Whole cell lysates of DHT stimulated *CWR*22Rν1 and C_4-2_ cells with/without MEM (40 μg/ml: 24h) were subjected to SDS-polyacrylamide gel electrophoresis, and effect of treatment was evaluated on AR and PSA protein levels. Densitometric analysis of immunoblots from three independent experiments was performed using Image J after normalizing to GAPDH; values plotted for each protein are shown in respective histograms. +*p<0.05 vs. DHT stimulated cells was considered statistically significant.
(TIF)

S7 Fig Effect of MEM treatment on tumor growth and apoptosis in a *CWR*22Rν1 xenograft mouse model. Whole cell lysates of tumor xenografts from animals treated with/without MEM were subjected to SDS-polyacrylamide gel electrophoresis. Equal loading was confirmed by reprobing with GAPDH. Densitometric analysis of immunoblots from three independent experiments was performed using Image J after normalizing to GAPDH; values plotted for each protein are shown in respective histograms. *p<0.05 and **p<0.01 vs. control were considered statistically significant.
(TIF)

S1 Pathologist Report Toxicity studies of MEM treated mice. Detailed report generated by pathologist after studying the tissues sections stained by H&E, of mice treated with DMSO/MEM.
(DOC)
